# Immunomodulation in Human Dendritic Cells Leads to Induction of Interferon-Gamma Production by *Leishmania donovani* Derived KMP-11 Antigen via Activation of NF-*κ*B in Indian Kala-Azar Patients

**DOI:** 10.1155/2014/947606

**Published:** 2014-01-22

**Authors:** Rajesh Chaudhary, Ajay Amit, Anupam Yadav, Anurag Singh, Vikash Kumar, S. K. Singh, Shyam Narayan, Vidyanand Rabidas, K. Pandey, Anil Kumar, Pradeep Das, Sanjiva Bimal

**Affiliations:** ^1^Rajendra Memorial Research Institute of Medical Sciences, Agamkuan, Patna, Bihar 800007, India; ^2^Division of Immunology, Rajendra Memorial Research Institute of Medical Sciences, Agamkuan, Patna, Bihar 800007, India

## Abstract

Dendritic cells (DCs) and macrophages (MΦs) are well-known antigen presenting cells with an ability to produce IL-12 which indicates that they have potential of directing acquired immunity toward a Th1-biased response. The aim of this study was to examine the effect of *Leishmania* specific KMP-11 antigen through comparison of immune responses after presentation by DCs and MΦs to T cells in Indian patients with VL. Patients with DCS and MΦs were directed against a purified *Leishmania donovani* antigen (KMP-11) and phytohaemagglutinin (PHA). The cytokines (IL-12, IL-10, and TGF-*β*) producing abilities of the DCs and MΦs against these antigens were determined by flow cytometry. The transcription factor (NF-*κ*B) and T-cell cytokine support (IFN-*γ*, IL-10), which could be significant in effector immune function, were also determined. Severe hindrance in the immune protection due to *Leishmania* parasites, as revealed by decreased expression of IL-12 and upregulation of IL-10 and TGF-*β* expression in the MΦs compared to DCs, occurred in VL patients. The production of IL-12 in response to *L. donovani* KMP-11 antigen was increased in DCs which was reduced in MΦs of VL patients. In contrast, the presentation of KMP-11 antigen by DCs to T-lymphocytes in VL patients significantly increased the IFN-*γ* produced by these immune cells, whereas the levels of IL-10 were significantly elevated after presentation of KMP-11antigen by MΦs. The VL patients were observed with severely dysfunctional MΦs in terms of NF-*κ*B activity that could be recovered only after stimulation of DCs with *L. donovani* KMP-11 antigen. Immunologically the better competitiveness of KMP-11 antigen through a dendritic cell delivery system may be used to revert T-cell anergy, and control strategy can be designed accordingly against kala-azar.

## 1. Introduction

Among the various forms of leishmaniasis, visceral leishmaniasis (VL) caused by *Leishmania donovani* (*L. donovani*) in the Indian subcontinent is the most severe and fatal if untreated. InVL, the causative agent, is transmitted by the phlebotomine sandfly to mammalian hosts, where they reside primarily within macrophages (MΦs) and dendritic cells (DCs). MΦs are well known as effectors of the innate immune system and are able to direct acquired immunity toward a Th1/Th2 biased response by their abilities to produce IL-12 and IL-10. DCs are the most potent type of the antigen-presenting cells (APC) and play a critical role in the initiation of immunity by producing soluble factors such as chemokines and cytokines [1]. InVL MΦs ingest promastigotes but these cells seem to synergies with parasite to facilitate infection [2–4]. Different studies have shown that, in addition to MΦs, infection of *Leishmania* parasite in DC has also been reported earlier [5, 6]. These cells as antigen-presenting cells (APCs) are able to induce a primary immune response and establishment of immunological memory [7]. *In vivo* infectivity of DC by *L. donovani* was also shown in mouse models [8]. Furthermore, different studies have shown that DC and MΦ are thought to distinguish different pathogens through the recognition of pathogen-associated molecular patterns (PAMP) via the expression of pattern recognition receptors (PRR) such as the Toll-like receptor family that decode the microbial surface proteins [9–11]. The outer membrane of *Leishmania* is covered by a dense glycocalyx consisting predominantly of lipophosphoglycan (LPG) [12]. Kinetoplastid Membrane Protein 11 (KMP-11) is a major surface protein which remains noncovalently associated with LPG complex especially in *L. donovani* species [13]. *In vitro* and *in vivo* studies using purified parasite protein have identified KMP-11 as a multifunctional immunogenic factor required for the protection from infection and there is widespread T-cell epitope conservation of this protein as well [14]. The roles ascribed to KMP-11 include reversal of T-cell anergy and upregulation of the expression of inducible nitric oxide synthase and synthesis of interleukin-12 (IL-12) in animal model [15, 16]. However, although such reports are encouraging, the efficacy may be variable between animals and human patients. Macrophages are preferred host for *Leishmania,* but these cells seem to synergies with parasite to facilitate infection [2–4] and because of this, there is a strong possibility for diminution of such effects of KMP-11 in infected MΦs in human VL cases. But its involvement in antigen presentation in the clinical scenario, especially in case of VL however, remains to be investigated. In the present study, we investigated whether monocyte-derived dendritic cells (moDCs) have different potential than MΦs to generate cytokines and drive CD4 Th1 cytokine expression after stimulation with a purified *L. donovani *protein (KMP-11) in the Indian VL patients.

## 2. Material and Methods

### 2.1. Expression, Isolation, and Purification of rKMP-11 Protein

To obtain the recombinant protein preparation from *Leishmania,* the plasmid (pQE-30) containing the 273 bp *L. donovani* specific KMP-11 gene which was 3.4 kb was cultured in Luria Broth suspension medium containing ampicillin (25 *μ*g/mL), kanamycin (100 *μ*g/mL) overnight at 37°C under 200 RPM in shaker incubator for 4-5 h. The recombinant protein was subsequently induced by Isopropyl *β*-D-1-thiogalactopyranoside (IPTG) (1 mM/mL) overnight in shaker incubator at 22°C and 200 RPM. The bacterial cells were harvested, pelleted (5000 RPM), and lysed in cell lysing solution (150 mM NaCl, 10 mM Tris HCl, 2% SDS; pH 8.0) in 1 : 4 ratio for 30 min at 4°C, and further ultrasonicated at 85% amplitude and 0.5-second pulses for 5 min. Following centrifugation (14000 RPM at 4°C), recombinant protein was purified on a Ni^+2^-NTA superflow column (Qiagen) according to the manufacturer's instructions. The protein in its denatured form was eluted in 8 M urea salt buffer with 250 mM imidazole and dialysed in PBS at pH 7.4. The protein expression was analysed by immunoblotting using mouse anti-KMP-11 Mab, clone L157 (GenWay, USA). Bacterial lipopolysaccharide (LPS) contamination in the recombinant protein (KMP-11) preparation was determined using the Limulus amoebocyte lysate (LAL) test (Thermo-Scientific, USA). A LPS contamination (0.11 *μ*g/mg of protein) was detected in the KMP-11 preparation. LPS in recombinant protein KMP-11 was completely removed by passing through polymyxin B-agarose column (Sigma, USA) according to the manufacturer's instructions and confirmed by LAL test. The recombinant KMP-11 protein was then stored at −80°C for further use [17].

### 2.2. Samples from VL Patients and Control

Peripheral-blood mononuclear cells (PBMCs) were obtained from buffy coats from age and gender matched VL patients and healthy donors using Ficoll-Hypaque (Pharmacia Biotech, Uppsala, Sweden) density gradient centrifugation at 800 ×g, 15 min at 20°C [18]. APCs (MΦs and moDCs) were taken from these healthy and *L. donovani* infected individuals and were stimulated with recombinant protein (KMP-11) prepared to look at the immunological response of the cells. These APCs were derived from 10 human patients with acute kala-azar (KA) in their pretreatment stage and 10 normal controls. Blood samples from KA patients were collected from the Department of the Clinical Medicine Unit, Rajendra Memorial Research Institute of Medical Sciences, Patna, Bihar, India. These KA patients were all male and of mixed age (ranging from 15 to 45 years) and were rK-39 and direct agglutination test positive but human immunodeficiency virus (HIV) negative. The parasite burden in splenic aspirates was determined as described previously by Chulay and Bryceson [19]. Each of the control subjects had no apparent history of VL and they did not reside in the VL endemic areas.

### 2.3. Generation of Macrophage (MΦs) and Monocyte-Derived Dendritic Cells (moDCs)

Heparinised samples of venous blood from patients and controls were used to procure APCs and PBMCs were isolated from Buffy coats using Ficoll-Hypaque density gradient centrifugation. Monocytes from PBMCs of KA patients were isolated by adherence of the cells in a plastic petri-dish and its purity was determined by FACS Calibur (Becton-Dickinson FACS-Calibur equipped with CellQuestPro Software, USA) of CD14, CD19, CD45, and CD3 expression [20], which were further cultured for another 72 h. Cell preparations were >92% MΦs and <0.5% T lymphocytes as assessed by fluorescence (anti-CD14 and anti-CD19 monoclonal antibodies, BD, USA) and size (FACS Calibur, BD, USA) [21]. The unfixed cells were stained with trypan blue which demonstrated that >95% cells were viable during incubation. DCs were obtained from monocytes after treatment with IL-4 (1000 U/mL) and granulocyte-macrophage colony stimulating factor (GM-CSF) (800 U/mL) on days 0, 3, and 6 in complete RPMI medium for 7 days. Immature DCs harvested on day 7 were further cultured for 48 h to differentiate in the presence of recombinant-Human TNF-*α* purified (20 ng/mL; Clone: MAb1, Isotype: Mouse IgG1, *κ*; eBioscience, Inc.). Viability of these DCs were found to be > 90% during incubation. The phenotypes of DC were determined in FACS by expression of CD1a, CD14, HLA DR, CD80, CD86, and CD83 expression. Antibody stained cells were evaluated using four-color FACS Calibur (Beckton Dickinson, USA) [22, 23]. The absence of endotoxins in DCs and MΦs was demonstrated by LAL test as discussed in the preceding section.

### 2.4. Intracellular Cytokine Produced from APCs

We initially examined the capacity of moDCs and MΦs to generate cytokines (IL-12, IL-10, and TGF-*β*) after stimulation with purified KMP-11 protein. In brief, to give an initial antigen pulsing, cells (APCs) were stimulated with fixed (2% formaldehyde) Ld promastigote antigen in responder (APCs) to stimulator (fixed Ld) ratio of 1 : 50 for 2 h at 37°C [24] and of them 1 × 10^6^ cells were cultured in 96-well round bottomed plates in the presence of purified KMP-11 protein (10 *μ*g/mL). Control cultures were set up in medium alone or medium containing phytohaemagglutinin (PHA) 10 *μ*g/mL. Intracytoplasmic cytokine level was detected on FACS-Calibur as previously described. Cells were cultured for 14 h followed by 4 h incubation with a protein transport inhibitor, brefeldin-A (1 *μ*g/mL). The harvested cells were consecutively coincubated with PE-conjugated anti-CD83 antibodies/anti-CD14-PE antibodies, cytofix/cytoperm solution, and FITC conjugated IL-10/IL-12/TGF-*β* (BD Pharmingen, USA) before each sample was resuspended in 500 *μ*L stain buffer. Samples were analysed on FACS-Calibur.

### 2.5. Cytokine Enzyme-Linked Immunosorbent Assay

To examine the relationship between the cytokine production profiles by the FACS based intracellular cytokine assay, after polyclonal stimulation with KMP-11, SLA, and PHA stimulation, we cultured representative DCs-T-cells and MΦs-T-cells cultured samples (1 × 10^6^ cells/mL) from patients and controls for 72 h. Cytokine levels (IL-12, IFN-*γ*, and IL-10) were measured in culture supernatants by sandwich ELISA kit (BD Pharmingen, San Diego, CA, USA).

### 2.6. Effect of KMP-11 Antigen on NF-*κ*B Production in moDCs and MΦs

moDCs or MΦs (1 × 10^6^) were suspended in 1 mL of RPMI-1640 medium and pulsed with formalin fixed *L. donovani* promastigotes in 24-well tissue culture plates for 14 h. The cells were then stimulated with KMP-11 antigen for 16 h at 37°C. Nucleic preparation was then obtained by incubating the washed (400 g, 5 min at room temperature) cells with 250 *μ*L of a solution containing trypsin, a spermine tetrahydrochloride detergent buffer (BD Pharmingen, San Diego, CA, USA) for 10 min at RT to digest cell membrane and to stabilize the nuclear chromosome. The cells were later treated with 200 *μ*L of a solution containing trypsin inhibitor and RNase buffer (BD Pharmingen, San Diego, CA, USA). The nuclei were incubated with PE-labelled anti-nuclear factor-*κ*B (anti-NF-*κ*B p65) antibody (Santa Cruz Biotechnology, Inc.). Washed cells were resuspended in 500 *μ*L of stain buffer and production of NF*-κ*B in moDCs and MΦs of patients and control samples was determined by FACS-Calibur.

In parallel experiments, 20–30 *μ*g of nuclear extract of moDCs and MΦs, either stimulated with KMP-11 or unstimulated, was separated by 12.5% polyacrylamide gel electrophoresis (PAGE) with sodium dodecyl sulphate (SDS). Separated proteins in the gel were transferred onto 0.22 *μ*m nitrocellulose membranes (Sigma Aldrich, USA) by an electroblot apparatus (Bio-Rad). The blot paper was then left for 2 h at RT before being washed thrice with PBS-T (PBS containing 0.1% Tween-20) and then soaked in 2% (IgG-free) BSA for 2 h at 37°C, to block any nonspecific binding sites. The blot paper was washed once again with PBS-T before being incubated for 2 h at 37°C with a 1 : 1000 dilution of the NF-*κ*B (Santa Cruz Biotechnology, Inc.). Unbound MAb was then removed by three washes with PBS-T before any bound antibody was labelled for 2 h at 37°C with avidin-horseradish-peroxidase conjugate used in 1 : 5000 (BD Biosciences, USA). After 5 washes, color was developed with diaminobenzidine (0.06% in 0.5 M citrate-saline, with 0.1% H_2_O_2_) for 15 min in the dark.

### 2.7. Cytokine Released from CD4+ T-Lymphocytes

Subsequent experiments were performed to look at the capacity of these two different APC subsets to drive CD4 T-cell cytokine response after stimulation with purified *L. donovani* protein (KMP-11) in VL patients and controls. In brief, 5 × 10^6^ autologous PBMCs were cocultured with stimulated or nonstimulated moDCs and MΦs from patients and controls. For this, the PBMCs were added to the wells with already primed MΦs or moDCs and cultured for 6 days with either medium alone or antigens of WHO reference strain *Leishmania* (20 : 1). The levels of expression of IFN-*γ* and IL-10 in CD4+ T cells of the patients were determined by using anti-CD4 antibodies and FITC labelled IFN-*γ*/IL-10 antibodies by FACS-Calibur. Remaining steps were the same as described in the preceding sections.

### 2.8. Statistical Analysis

All data were expressed as mean ± SE (standard error of the mean). One way analysis of variance with Tukey post hoc test was carried out using GraphPad Prism5, USA, software. A value of significance *P* < 0.05 was considered statistically significant.

## 3. Results

### 3.1. Characterization of KMP-11

Results on SDS polyacrylamide gel electrophoresis of KMP-11 purified recombinant protein and the localization of KMP-11 protein after immunoblotting with anti-KMP-11 antibody are shown in Figure 1. The extraction of KMP-11 protein was achieved by Ni^2+^-NTA immobilized column chromatography. The bound protein was eluted in the presence of imidazole and later subjected to 12.5% SDS-PAGE (Figure 1(a)). The anti-KMP-11 mAbs were later used in immunoblots on SDS-PAGE separated KMP-11 proteins from *Leishmania* spp. which were previously purified by Ni^2+^-NTA affinity column. The mAbs detected bands of approximately 11 KDa (Figure 1(b)).

### 3.2. Phenotypic Characterization of DCs

Human PBMCs were cultured in complete RPMI-1640 medium containing GM-CSF and IL-4 for 7 days followed by 2-day maturation in the presence of recombinant-human-TNF-*α*. Phenotypic characterization of mature DCs was demonstrated for expression of costimulatory molecules (CD80, CD83, and CD86) in VL cases.  Figure 2(a) shows that large cells were gated and Figure 2(b) (B1-B2) showing differentially expressed molecule CD83 (B1) and HLA-DR (B2). The expression was done on at least 3 separate patients. The differentially expressed molecule is CD1a positive.  Figure 2(c) shows mature DCs showing a lesser percentage of CD1a positivity in CD14 and CD1a double stained cells.  Figure 2(d) (D1-D2) shows inverted microscopic picture of immature and mature DCs.  Figure 2(e) shows mature MΦs showing a greater percentage of CD14+ cells than CD19+ cells after 72 h culture.

### 3.3. Cytokine Production by KMP-11 Stimulated MΦs and moDCs

To understand APCs related differences, cytokine immune cell response was examined in moDCs that expressed CD83, CD86, CD80, and HLA-DR and MΦs that expressed CD14 in response to purified *L. donovani * antigen (KMP-11) with flow cytometry (Figures 3 and 4). The initial parameters examined were IL-12, which is required for host protection, and IL-10 and TGF-*β*, known to induce strong immunosuppression following *L. donovani* infection.

The results revealed higher percentage of IL-10 and TGF-*β* in patients with VL compared with the healthy controls (*P* < 0.001). However, after activation of DCs with *Leishmania* KMP-11 antigen expression of IL-10 and TGF-*β* remained low whereas expression level of IL-10 and TGF-*β* by MΦ remained higher than in DCs (*P* < 0.001). These results indicate that *Leishmania* did not influence the triggering of immune-suppression factors, especially during presentation of *Leishmania* KMP-11 antigen to DCs in VL (*P* < 0.05) compared to unstimulated. Indeed, VL participants presented with greater upliftment of IL-12 expression in DCs after activation with KMP-11 antigen compared with MΦ results and the control group (*P* < 0.001).

### 3.4. *Leishmania* Contributes to Inhibiting NF-*κ*B Signalling in MΦs Which Are However Upregulated by KMP-11 Antigen in moDCs in VL Patients

The differences in the production of IL-12 by moDCs and MΦs elicited by KMP-11 antigen prompted us to examine the activation of the NF-*κ*B by KMP-11 antigen. As illustrated in Figure 5, many striking differences were observed in moDCs and MΦs with regard to the NF-*κ*B activation in the VL patients. In general, it was observed that *Leishmania *contributed to inhibiting NF-*κ*B signalling, the evidence of which was more predominant in MΦs rather than moDCs of the VL patients. A significant increase in NF-*κ*B pattern was observed in MΦs and DCs when stimulated with KMP-11 and PHA in comparison with their respective un-stimulated (VL and ctrl.) populations (*P* < 0.001). However, we observed a high expression of NF-*κ*B in KMP-11 or PHA stimulated DCs in comparison to KMP-11 or PHA stimulated MΦs. NF-*κ*B production in DCs increased after stimulation with KMP-11 antigen about 11.22-fold (*P* < 0.001) higher from base value (*ex vivo*) in VL patients. Comparatively, there was observed significantly lower (3.2-fold, *P* < 0.05) ability of MΦs to produce NF-*κ*B after the KMP-11 antigen stimulation from base value. When compared between APCs, ability of MΦs to produce NF-*κ*B was lower (2.1-fold, *P* < 0.001) in KMP-11 stimulated group than the DCs in patients. A significant difference was observed among VL patients (*P* < 0.001) and control groups (*P* < 0.01) of MΦ and DC populations, respectively. There was no significant difference observed between VL and Ctrl. groups of MΦs and DCs in different groups, respectively. However VL patients (un-stimulated) have shown 4.92-fold and 1.30-fold increase in NF-*κ*B pattern in MΦs and DCs population, respectively (Figure 5).

### 3.5. Interaction of DCs with CD4+ T Cells Contribute to Intense IFN-*γ* Production in Response to KMP-11 Antigen

We finally validated the potency of DCs in priming and directing CD4 T cell cytokine immune response to KMP-11 in VL cases (Table 1). There was absence of *Leishmania *specific T cell response in healthy control T cells. The IFN-*γ* and IL-10 ranges for the healthy control T cells in the absence or presence of costimulation were lower. In fact, no difference was seen comparing IFN-*γ* and IL-10 range before and after costimulation for moDCs and MΦs in the control. On the other hand, considerable differences were observed in these APCs at the level of costimulation through KMP-11 antigen compared to the corresponding values obtained in the absence of costimulation in VL patients. In general the IFN-*γ* produced during the interaction of DCs with CD4+ T cells was 7.63-fold higher in response to KMP-11 than *ex vivo* value (*P* < 0.001). When the MΦs presented the KMP-11 antigen, IFN-*γ* production in the same CD4+ T cells was only 2.49-fold greater in response to KMP-11 than *ex vivo* value (*P* > 0.05). On the other hand, the presentation of KMP-11 antigen by MΦs induced 2.41-fold IL-10 in the T cells of VL patients compared to when DCs presented the KMP-11 antigen (*P* < 0.001). The difference between moDCs and MΦs became obvious with the finding that IL-10 produced during the interaction of MΦs with T-cells were 6.19-fold higher than control (*P* < 0.001) whereas CD4 cells during an interaction with moDCs yielded about 1.72-fold lower IL-10 response to KMP-11 antigen of *L. donovani.*

The cytokine polarization index (Log_e_ IFN-*γ*: Log_e_ IL-10) (Figure 6) was observed to be more polarized towards IFN-*γ* after stimulation of MΦs and DCs with KMP-11 in VL patients compared to controls. The comparison revealed that this polarization was more towards IFN-*γ* after stimulation of DCs with KMP-11 protein.

### 3.6. Secreted Levels of IL-12, IFN-*γ*, and IL-12 in Culture Supernatants

Since the supernatants of cultures of all the samples were not stored, in the representative supernatants of the cultures of 3 VL patients and 3 healthy controls, secreted levels of IL-12, IFN-*γ*, and IL-12 were estimated by ELISA. Levels of IL-12 and IFN-*γ* were high after presentation of *L. donovani* specific antigen KMP-11 by DCs to T cells in VL patients. On the contrary, levels of IL-10 were high when KMP-11 antigen of *L. donovani* was delivered by MΦs to T cells in the VL patients compared with DCs-T counterparts and healthy controls (Table 2).

## 4. Discussion

The present study successfully demonstrates that *L. donovani* specific KMP-11 antigen can act to promote host protective immune response during chronic phase of infection with *L. donovani*. Furthermore, by comparing the role of DCs and MΦs in the presence of this *L. donovani* specific antigen during the chronic phage of VL, we could show that whereas both DCs and MΦs contribute to suppress host protective immune response *ex vivo,* it was this KMP-11 antigen which was capable of promoting the activation of DCs in VL patients that produced IL-12.

There were two reasons why KMP-11 was chosen as the testing antigen. Firstly, lipophosphoglycan linked KMP-11 is the major protein on the promastigote surface which plays a key role in immunity against this parasite [14, 25, 26]. The induction of IFN-*γ* is critical for resistance and cure in all forms of leishmaniasis [27, 28]. In this context, 30 peptides of KMP-11 antigen were identified from sequence analysis which reportedly triggered IFN-*γ* secretion [29]. Unlike previous studies assessing the role of KMP-11 antigen in human blood samples of VL patient, sustained population of DCs during ongoing infection was required in the present study. In humans, at least two types of DCs are known to exist such as plasmacytoid (pDC) and myeloid (mDC). The pDCs depend on IL-3 and elicit a Th2 type response [30]. GM-CSF and IL-4 appear to be instrumental in generating mDCs from peripheral blood monocytes. The role of IL-4 has been implicated to suppress the generation of MΦs [31] and yielding CD1a myeloid DC subset, which under the influence of CD83 promotes MHC Class II and co-stimulatory molecules [32] to induce a more mature phenotype of CD83+ DCs. Several other previous studies also showed that DC could develop from CD14+ blood monocytes cultured with GM-CSF and IL-4 [33]. We obtained DCs from human peripheral blood. It is clearly mentioned that mature DCs undergo cell surface phenotypic changes that include the expression of co-stimulatory molecules, such as MHC Class II molecule, CD80, CD86, and CD40. They also express CD83 [34] as such expression of co-stimulatory molecules. Accordingly DCs were derived from peripheral blood monocytes cultured in the presence of GM-CSF and IL-4 (7 days). They were induced to maturity by TNF-*α* added on day 7 for another 48 h. Expression of CD80, CD86, CD83, and HLA-DR was determined on mature DCs. By incorporating this information into our study, we could transform a high percentage of CD1a^dim⁡^DC by stimulation with TNF-*α* in peripheral blood monocytes of patients infected with *L. donovani* similar to the efficacy reported for DC generation in VL patients [35]. A strong immune-suppression is a characteristic feature of *L. donovani* infection which encourages the parasite to impair free radical (super oxide and nitric oxide) generation [36] and IL-12- a host protective cytokine production [37]. In experimental* Leishmania *infection, IL-12 is also required for the induction of Th1-related chemokines such as XCL1 (also known as lymphotactin) and IFN-inducible protein 10 (also known as CXCL10 or IP-10) which are associated with immune protection [38]. However, usually, the disease promoting cytokines, TGF-*β* and IL-10, are enhanced in *L. donovani* infection [39, 40]. Surprisingly, even a KMP-11 stimulation given to MΦs could not augment adequate IL-12 production in VL patients. Earlier studies also suggest that *Leishmania *has the ability to suppress IL-12 production in MΦs [2, 4, 41]. Of note, in spite of stimulation, TGF-*β* and IL-10 were observed to increase in MΦs which suggested that all parameters of host resistance that we measured were suppressed in MΦs even after stimulation with KMP-11 antigen. Importantly we could not distinguish much between the effects *ex vivo* and after KMP-11 stimulation. An important characteristic feature of VL is production of the immuno-regulatory cytokine IL-10 and targeting of IL-10 signalling has been identified as a potential therapeutic strategy [24, 42–44]. IL-10 suppresses IFN-*γ* induced NO production [45]; hence the increase of IL-10 expressing MΦs may itself underlie the suppression in MΦs due to *Leishmania* infection. In contrast, the cytokine response profile triggered by KMP-11 antigen in DCs had differential characteristics such as an increase in IL-12 production concomitantly with a marked decrease in TGF-*β* and IL-10 production.

During the study on differential effects of APCs on T cells against the KMP-11 antigen, we provided a long incubation to T cells exposed *Leishmania* KMP-11 antigen anticipating that they had previously been sensitized *Leishmania* from MΦs and it would be difficult to observe the effect of *Leishmania* KMP-11 antigen presented via DCs to the T cells in a shorter period. Reiner et al. (1990) [46] showed that incubation time did not affect the usual pattern of cytokine response. However, in this earlier study, parasite delivery was done by MΦs only while we attempted to sensitize the T cells with *Leishmania* KMP-11 antigen from two different sources.

Unlike previous data showing an impact of KMP-11 antigen in the stimulation of effector IFN-*γ* producing CD4 cells, the stimulation of T cells after presentation of KMP-11 antigen by MΦs during infection did not significantly affect IFN-*γ* production by CD4+ T cells, suggesting that testing the efficiencies of an immunogenic candidate via delivery through MΦs may suffer as the MΦs could not be essential for the maintenance of effector T-cell response. However, our data were in contrast when we delivered the KMP-11 antigen to T cells via DCs showing that the presentation of the same antigen by DCs during established infection with *L. donovani* resulted in a significant increase in IFN-*γ* production by CD4+ T cells. The chronic *L. donovani* infection is associated with expansion of CD4+ T cells that express IL-10. The further analysis made here indicates that, during *L. donovani* infection, KMP-11 antigen decreases IL-10-producing CD4+ T cells after its delivery via DCs which was more pronounced through DCs compared to the MΦs. Thus, though KMP-11 antigen was an effective immunogen, it required providing optimum immune-stimulatory effects only when delivered to T cells via DCs. Hence, the requirement for KMP-11 antigen to maintain T-cell IFN-*γ* production would appear to be more protection-specific, when presented by DCs rather than MΦs.

MΦs have multiple functions; they serve as host cells for parasite replication, as antigen-presenting cells, and as a source of cytokines modulating the T-cell mediated immune response. Moreover, after appropriate activation by Th1 cells, they serve as effector cells for *Leishmania* killing. Inferential results suggest that *Leishmania* abrogates the abilities of MΦs to abruptly disturb emergence of a Th1-like cell response during *L. donovani* infection. The data generated in this study also have hinted toward the lesser potential of MΦs as APCs during VL in humans. This might be due to inadequate expression of MHC Class II molecules on MΦs required for the induction of effective immunity. This speculation is well in accordance with the findings of a previous study in *L. major *suggesting MΦ antigen presentation may not be required for effector T-cell function [47].

Nevertheless, KMP-11 primed moDCs generated adequate IL-12 which reflected that it can have a specific effect on T-cell response that was severely impeded in KMP-11 stimulated MΦs of the same patients. Reports on infectivity of *L. donovani* are available [6] and DCs have also been observed to produce IL-12 after infection with *L. major* [48] and *L. amazonensis* [49].

The differential production of IL-12 between MΦs and DCs was observed mainly due to differences in NF-*κ*B production after the presentation of *L. donovani* KMP-11 antigen. This difference may offer distinct signals to immune cells that can affect differentiation of CD4+ T cells to Th1 or Th2. In support of this possibility, it is known that these cells require NF-*κ*B support for maturation [50]. Moreover, the signalling initiated by TNF receptor associated factor 2, 3 (TRAF 2-3) at cholesterol rich membrane rafts on the plasma membrane of DCs leads to p38 MAP kinase phosphorylation for CD40 mediated IL-12 production of different types of *Leishmania *[51, 52]. The src family protein kinase, Lyn, is reported to simultaneously activate the ERK pathway during the process [51]. Further, the NF-*κ*B has been shown to be required for the production of IL-12 and IFN-*γ* as well as inducible nitric oxide synthase (iNOs) [53–56].

This extent of formidable immunological changes in moDCs was hitherto not observed to occur in MΦs, suggestive of the importance of APCs in judging the immunogenic potential of KMP-11 as a mean to achieve a protective immune response in VL patients. Thus, we found that the KMP-11 antigen of *L. donovani* had the ability to produce IL-10 and TGF-*β* in MΦs and IL-12 in DCs in VL patients. Such alterations in cytokine production in response to KMP-11 antigen which we have observed in this study can contribute to bias the immune response which may be important for the outcome of the disease.

## Figures and Tables

**Figure 1:** (a) SDS polyacrylamide gel electrophoresis of *L. donovani* of KMP-11 purified recombinant protein and (b) western blot analysis. (a) SDS polyacrylamide gel electrophoresis of *L. donovani* of KMP-11 purified recombinant protein. Coomassie brilliant blue staining Lane 1 Marker, Lane 2 CP- Crude Protein, Lane 3 E1 (eluted protein after first washing), Lane 4 E2 (eluted protein after the second washing), Lane 5 E3 (eluted protein after the third washing), Lane 6 F1, Lane 7 F2, Lane 8 F3 (Lane 6-7 protein fraction of KMP-11), and F3 fraction in Lane 8 show the KMP-11 recombinant protein. (b) KMP-11 recombinant protein purified by affinity chromatography, transferred on nitrocellulose paper, and probed with anti-KMP-11 antibody. The arrow indicates the localization of KMP-11 protein. The asterisks show the dimeric and trimeric forms of the KMP-11 protein.

**Figure 2:** Phenotypic characterization of mature dendritic cells for expression of costimulatory molecules (CD80, CD83, and CD86) in VL cases. Maturation was induced by 7-days stimulation of DC with TNF-*α* for 48 hours. (a) Large cells were gated. (b) (B1-B2) The differentially expressed molecule is CD83 (B1) and HLA-DR (B2). The expression was done on at least 3 separate patients. The differentially expressed molecule is CD1a. (c) Mature DCs showing a lesser percentage of CD1a positivity in CD14 and CD1a double stained cells. (d) (D1-D2) Inverted microscopic picture of immature and mature DCs. (e) Mature macrophage showing a greater percentage of CD14+ cells and a lesser percentage of CD19+ cells after 72 h culture.

**Figure 3:** (a) IL-12 release by MΦ and moDC after KMP-11 and PHA stimulation. (a) Comparison of cytokine production by APCs after costimulation by KMP-11. 1 × 10^6^/mL of either CD14+ MΦ or CD83+ moDCs was stimulated with KMP-11 (10 *μ*g/mL) and PHA (10 *μ*g) for 16 h. Harvested cells were consecutively coincubated with Bref-A (1 *μ*g/mL), surface CD-4 (PE)/CD-83 (PE) antibodies, and cytofix/Perm solution before cytoplasmic staining with FITC for IL-12 and acquired and analyzed on FACS-calibur. Values were expressed in mean ± SEM. Each sample was run in duplicate. ***P < 0.001 versus VL-MΦ; ^###^ *P* < 0.001 versus VL-DC; ^∧∧∧^ *P* < 0.001 versus Ctrl-DC; ^@^ *P* < 0.05 versus VL-MΦ-KMP-11 and ^$$$^ *P* < 0.001 versus respective MΦ and DC groups; and ^+^ *P* < 0.05 between VL-DC-KMP-11 and Ctrl-DC-KMP-11 groups. (b) Representative dot plot for the intracellular staining of IL-12 in MΦs and DCs of VL patients.

**Figure 4:** Flow cytometry analysis on reversal of immune-suppression in moDCs in response to *L. donovani* antigen after stimulation of KMP-11. (a)-(b) Comparison of cytokine production by APCs after costimulation by KMP-11. 1 × 10^6^/mL of either CD14+ MΦ or CD83+ moDCs was stimulated with KMP-11 (10 *μ*g/mL) and PHA (10 *μ*g) for 16 h. Harvested cells were consecutively coincubated with Bref-A (1 *μ*g/mL), surface CD-4 (PE)/CD-83 (PE) antibodies, and cytofix/Perm solution before cytoplasmic staining with FITC for IL-10 and TGF-*β* and acquired and analyzed on FACS-calibur. Values were expressed in mean ± SEM. Each sample was run in duplicate. ***P < 0.001 versus VL-MΦ; ^#^ *P* < 0.05, ^###^ *P* < 0.001 versus VL-DC; ^aaa^ *P* < 0.001 versus Ctrl-MΦ; ^@@@^ *P* < 0.001 versus VL-MΦ-KMP-11; ^bbb^ *P* < 0.001 versus VL-DC-KMP-11; ^cc^ *P* < 0.01, ^ccc^ *P* < 0.001 versus Ctrl-KMP-11; ^$^ *P* < 0.05,  ^$$$^ *P* < 0.001 versus respective MΦ and DC groups; and ^+++^ *P* < 0.001 between respective VL-DC and Ctrl-DC groups. (c) Representative dot plot for the intracellular staining of IL-10 in MΦs and DCs of VL patients.

**Figure 5:** Differential NF-*κ*B pattern after stimulation with KMP-11 in APCs of VL patients and healthy controls. The capacity of moDCs and MΦs for the activation of NF-*κ*B was compared through intracellular staining using fluorescent conjugated anti-NF-*κ*B antibodies on flow cytometry. Following stimulations (KMP-11 and PHA), cells were harvested and then incubated with PE-anti-p65 NF-*κ*B antibodies, acquired and analyzed on FACS Calibur. Total amount of NF-*κ*B was produced by MΦ and moDC stimulated and unstimulated with rKMP-11 evaluated through FACS calibur. Immunoblotting of VL MΦ and VL DCs (insert, Figure 5) with NF-*κ*B antibody shows that KMP-11 triggered significant phosphorylation of a protein migrating at 65 kDa of NF-*κ*B. There was no significant difference observed between DC-Ctrl and VL-DC of respective groups. *P < 0.05, ***P < 0.001 versus VL-MΦ; ^###^ *P* < 0.001 versus VL-DC; ^a^ *P* < 0.05, ^aaa^ *P* < 0.001 versus Ctrl-MΦ; ^∧∧∧^ *P* < 0.001 versus Ctrl-DC; ^@^ *P* < 0.05 versus VL-MΦ-KMP-11 and ^$$^ *P* < 0.01,  ^$$$^ *P* < 0.001 versus respective MΦ and DC groups.

**Figure 6:** Cytokine polarization index after exposure of macrophages and moDCs to KMP-11 and subsequent coculture with T cells in VL patients and healthy controls. Cytokine polarization index after exposure of MΦs and moDCs to KMP-11 and subsequent co-culturing with T cells in VL patients. The index was obtained after calculating the ratio of log⁡_e_ IFN-*γ*: log⁡_e_ IL-10, based on FACS Calibur using CellQuest Pro software.

**Table 1:** Cytokine profile of CD4+ T-cell lymphocytes differentiated in response to stimulation with *L.donovani* specific KMP-11 antigen.

Source of APCs	Cytokines	Frequency of cytokine producing CD4+ T cells obtained after stimulation with different *Leishmania* antigen	
		*Ex vivo *	KMP-11
Macrophage			
Active VL (*n* = 10)	IFN-*γ*	2.765 ± 0.3928	6.88 ± 1.244**
	IL-10	4.42 ± 0.5656	27.4 ± 3.512
Healthy control (*n* = 10)	IFN-*γ*	2.85 ± 0.4606	3.08 ± 0.3467
	IL-10	1.89 ± 0.2023	1.73 ± 0.1322
Monocyte-derived dendritic cell			
Active VL (*n* = 10)	IFN-*γ*	2.29 ± 0.2415	17.48 ± 2.17**
	IL-10	19.51 ± 1.608	11.34 ± 0.916
Healthy control (*n* = 10)	IFN-*γ*	2.98 ± 0.5026	3.58 ± 0.432
	IL-10	1.97 ± 0.0928	1.73 ± 0.144

(i) Mean ± standard error.

(ii) These values came from a total lymphocyte gate (R1).

(iii) Frequencies after 5 days of culture with the indicated antigen (KMP: 10 *μ*g/mL) and PHA (10 *μ*g/mL).

(iv) Significantly different from the frequency *ex vivo* using student's *t*-test with comparison of all pairs and a *P* value of <0.05  *ex vivo* and KMP-11 antigen (**).

**Table 2:** Secreted levels of IL-12, IFN-*γ*, and IL-10 in the culture supernatants after differential stimulation and antigen presentation in VL patients and controls.

Subjects	IL-12 (pg/mL)		IFN-*γ* (pg/mL)		IL-10 (pg/mL)	
	DCs-T	MΦ-T	DCs-T	MΦ-T	DCs-T	MΦ-T
VL						
SLA	32.3 ± 4.015*	18.5 ± 1.57	94.5 ± 7.067	54.6 ± 4.45	142.5 ± 5.202	213 ± 17.22
KMP-11	61.8 ± 8.113	52.6 ± 4.605	325.3 ± 20.42	207.1 ± 12.65	122.7 ± 10.66	160.0 ± 11.72
PHA	55.4 ± 3.166	55.7 ± 4.138	270.7 ± 43.36	210.0 ± 7.638	190.9 ± 18.27	320.3 ± 16.39
Healthy-Ctrl.						
SLA	56 ± 9.48	50 ± 12.54	124.5 ± 20.46	89.9 ± 4.378	20.1 ± 2.597	24.4 ± 2.61
KMP-11	70 ± 11.4	66 ± 9.803	188.9 ± 17.91	110.55 ± 11.70	9.2 ± 0.6727	12.7 ± 1.453
PHA	120 ± 14.39	110 ± 7.855	157.8 ± 15.75	122.30 ± 15.74	13.2 ± 1.012	16.5 ± 0.9539

*Mean ± standard error.
